# Beclin-1-independent autophagy positively regulates internal ribosomal entry site-dependent translation of hypoxia-inducible factor 1α under nutrient deprivation

**DOI:** 10.18632/oncotarget.2265

**Published:** 2014-07-26

**Authors:** Ching-An Wu, Duen-Yi Huang, Wan-Wan Lin

**Affiliations:** ^1^ Department of Pharmacology, College of Medicine, National Taiwan University, Taipei, Taiwan; ^2^ Graduate Institute of Medical Sciences, Taipei Medical University, Taipei, Taiwan

**Keywords:** nutrient deprivation, Beclin-1-independent autophagy, HIF-1α, IRES, hypoxia, ATG5-independent autophagy

## Abstract

Hypoxia has been shown to induce hypoxia-inducible factor-1alpha (HIF-1α) expression to support many cellular changes required for tumor growth and metastasis. In addition to hypoxia, nutrient deprivation is another stress condition widely existing in solid tumors due to the poor blood supply. Our data showed that nutrient deprivation induces a significant HIF-1α protein expression and potentiates the HIF-1α responses of hypoxia and CoCl_2_. This effect is not because of enhancement of HIF-1α stability or transcription. Rather we found it is through the cap-independent but internal ribosome entry site (IRES)-dependent translation. Notably inhibition of autophagy by si-ATG5, 3-methyladenine and chloroquine, but not si-Beclin-1, significantly reverses nutrient deprivation-induced HIF-1α responses. Furthermore, it is interesting to note the contribution of IRES activation for hypoxia-induced HIF-1α expression, however, different from nutrient starvation, si-Beclin 1 but not si-ATG5 can inhibit hypoxia-induced HIF-1α IRES activation and protein expression. Taken together, we for the first time highlight a link from alternative autophagy to cap-independent protein translation of HIF-1α under two unique stress conditions. We demonstrate Beclin 1-independent autophagy is involved to positively regulate nutrient deprivation induced-HIF-1α IRES activity and protein expression, while ATG5-independent autophagy is involved in the HIF-1 IRES activation caused by hypoxia.

## INTRODUCTION

Due to insufficiency of blood supply, hypoxia and starvation are two common features in solid tumors [1-5]. To cope with hypoxia and to maintain energy requirement, higher organisms have developed numerous adaptive responses to stimulate angiogenesis, glycolysis, and erythropoiesis [1, 3]. Many of these responses are mediated by hypoxia-inducible factor 1α (HIF-1α), whose stability and activity are regulated by oxygen. When hydroxylated by HIF-1-prolyl hydroxylase, HIF-1α is ubiquitinated by von Hippel-Lindau protein and then degraded by proteasome [6, 7]. Since hydroxylation is oxygen dependent, HIF-1α becomes stabilized and activated under hypoxic conditions.

Contrary to hypoxia, HIF-1α induced by various growth factors [8], cytokines [9], vascular hormones [10] and viral proteins [11] under normoxia condition are through enhancement of the HIF-1α protein translation. There are two basic mechanisms of initiating translation. One is cap-dependent, and the other is cap-independent. Cap-dependent translation is controlled by mTOR signaling which releases initiation factor eIF4E from 4E-BP1. An alternative route of translation is mediated by cap-independent activation via internal ribosome entry site (IRES). In contrast to cap-dependent translation which recruits translational complex to m^7^G cap structure at the 5′-end, IRES activation directly recruits 40S ribosomal subunit to the vicinity of the initiation codon [12]. In the case of HIF-1α, hypoxia, serum withdrawal [13] and tumor necrosis factor-alpha (TNF-a) [14] have been shown to induce HIF-1α IRES activity, however, the underlying mechanisms are still unclear.

Autophagy is a self-eating process which is highly conserved from yeast to mammals. During starvation, autophagy is induced to recycle cellular components to produce amino acids and fatty acids which serve as materials for mitochondrial energy production. There are different types of autophagy, including microautophagy, macroautophagy and chaperone-mediated autophagy (CMA) [15]. Of them, macroautophagy is the major process to recycle cytosolic proteins and organelles to provide energy under nutrient starvation. Macroautophagy is formed by multistep processes controlled by proteins termed autophagy-related (ATG) proteins [16]. The formation of the phagophore requires the class III phosphatidylinositol 3-kinase (PI3K), also known as Vps34 that forms a complex with Beclin 1. Apart from conventional macroautophagy, two alternative macroautophagy pathways respectively independent of ATG5/ATG7 and Beclin 1 have been described [17-21]. In mouse embryonic fibroblasts autophagy can be induced by cytotoxic stressor etoposide and starvation independent of ATG5, ATG7 or LC3-II accumulation. However, it was regulated by class III PI3K and Beclin 1 [18]. On the other hand, resveratrol, neutotoxin 1-methyl-4-phenylpyridinium (MPP^+^), arsenic trioxide, staurosporine and inhibitor of Bcl-X_L_/Bcl-2 can induce non-canonical macroautophagy which is class III PI3K- or Beclin 1-independent, but depends on ATG7 and LC3-II accumulation [20, 22-25].

In addition to proteasome, some evidence shows that HIF-1α is also degraded through autophagy-dependent pathway [26-28]. 15-Deoxy-delta (12,14)-prostaglandin-J_2_ induced HIF-1α accumulation by an inhibition of lysosome activity [26]. Inhibition of lysosome activity by bafilomycin A1, chloroquine or ammonium chloride induced HIF-1α accumulation in HeLa and Hep3B cells [27]. Furthermore, it has been demonstrated that HIF-1α is degraded through CMA-dependent pathway. 6-Aminonicotinamide, a commonly used activator of CMA, inhibits hypoxia-induced HIF-1 accumulation and overexpression of Hsc70 or LAMP2A, two CMA-dependent molecules capable of association with HIF-1α, decreased hypoxia-induced HIF-1α level [27]. Although CMA mediates HIF-1α degradation, one of their results showing that silence of ATG6 abolished hypoxia-induced HIF-1α accumulation raises the possibility that macroautophagy might positively regulate HIF-1α expression [27].

Starvation is another feature of solid tumors, however, compared to hypoxia the role of starvation in tumorigenesis still remains elusive. Our previous study demonstrated that nutrient-deprivation drives cancer cells to utilize glycolysis to produce ATP, also known as Warburg effect, and this action is through a novel mechanism involving ROS/AMPK-dependent activation of PDK [29]. In the present study, we tried to elucidate the effect of nutrient deprivation on HIF-1α accumulation in cancer cells and the underlying molecular mechanism. Therefore, we used Hank's buffered salt solution (HBSS) as a starvation model and found that Beclin 1-independent macroautophagy positively regulates nutrient deprivation-induced HIF-1α IRES-dependent translation pathway in HeLa cells.

## RESULTS

### HBSS induces HIF-1α expression and potentiates the HIF-1α responses of hypoxia and CoCl_2_

To understand the effect of nutrient deprivation on HIF-1α expression, the medium HBSS containing 5 mM glucose in the absence of 10% FBS was used as a starvation model to treat different cancer cell lines. As shown in Fig. 1A, HBSS significantly induced HIF-1α expression around 1 h treatment and sustained this effect over 5 h in HeLa cells. Considering the cell type-specificity of this effect, we tested various cancer and normal cell types. We found that HBSS still can increase HIF-1α expression in A431 and A375 cancer cells as well as the primary HUVEC (Fig. 1A). To further understand what nutrient component(s) deficiency is involved in the HBSS-induced HIF-1α expression, we supplemented glucose, amino acids or FBS in HBSS. As a result shown in Fig. 1B, we found that 25 mM glucose had no significant effect on HBSS-induced HIF-1α expression, while 10% FBS totally reversed HBSS-induced HIF-1α expression. Among the 5 amino acids (glutamine, leucine, arginine, histidine and cysteine) tested, which have been studied for nutrient deprivation [30-34], only cysteine, but not the combination of glutamine, leucine, arginine and histidine, significantly inhibited HBSS-induced HIF-1α expression (Fig. 1B). To test the effect of HBSS with other inducers on HIF-1α expression, HBSS was co-treated with hypoxia or CoCl_2_. As shown in Figs. 1C and 1D, the extent of HIF-1α expression induced by HBSS was similar to that under CoCl_2_ treatment, but is much less than that induced by hypoxia. Interestingly HBSS showed synergistic interaction with CoCl_2_ and hypoxia, suggesting that nutrient deprivation-induced HIF-1α expression is resulting from a mechanism different from CoCl_2_ and hypoxia.

**Figure 1:** HBSS induces HIF-1α expression and potentiates the HIF-1α responses of hypoxia and CoCl_2_ (A) HeLa, A431, A375 and HUVEC were treated with HBSS. At indicated time points, cell lysates were evaluated for the HIF-1 protein level. (B) HeLa cells were treated with HBSS for the indicated time periods, either in the presence or absence of four amino acids (4 mM glutamine, 0.8 mM leucine, 0.4 mM arginine, 0.2 mM histidine), glucose (25 mM), cysteine (0.2 mM) or 10% FBS. (C, D) HeLa cells were treated with HBSS for the indicated time periods, either in the presence or absence of hypoxia (C) or 200 μM CoCl_2_ (D). Total cell lysates were collected and subjected to Western blot analysis.

### HBSS enhances HIF-1α expression through IRES-dependent translation

To understand HBSS-induced HIF-1α expression through regulating transcriptional, translational and/or protein stability levels, different experiments were conducted. In the aspect of transcription, we found that HBSS has no effect on HIF-1α mRNA expression within 4 h (Fig. 2A). We conclude that HBSS-induced HIF-1α expression is not at transcriptional level. Next, we used cycloheximide (CHX), a general translation inhibitor, to determine if HBSS-induced HIF-1α expression is via affecting protein stability. After induction of HIF-1α by HBSS treatment for 4 h, HBSS was changed to complete DMEM with 10% FBS or remained in HBSS with or without CHX, and the HIF-1α protein degradation was determined. As shown in Fig. 2B, the HIF-1α protein degradation rate measured in complete DMEM media regardless of CHX treatment or not was similar, i.e. around 5 min of half-life. This result suggests that the protein degradation through proteasome system rather than protein synthesis process plays immediate and almost the major role in controlling HIF-1α protein expression. In cells with HBSS replacement and sustained HIF-1α expression, CHX treatment also rapidly led to protein degradation by 56% at 5 min, suggesting that HBSS-induced HIF-1α expression in major does not result from protein stabilization. To understand if HBSS-induced HIF-1α expression is through HIF-1α protein newly synthesis, de novo translation was conducted by [^35^S]methionine labeling. As shown in Fig. 2C, HBSS can enhance de novo HIF-1α translation. Similarly CoCl_2_ exerts this action as previously reported [35]. To directly demonstrate the ability of HBSS to enhance HIF-1α translation, the relative associations of HIF-1α mRNA with the polysomal and nonpolysomal fractions were determined. As shown in Fig. 2D, HBSS enhanced HIF-1α mRNA binding to polysome by 20%, while hypoxia has no significant effect as previously reported [13].

**Figure 2:** HBSS enhances HIF-1α expression through IRES-dependent translation (A) HeLa cells were treated with HBSS. At indicated time points cells were collected and HIF-1α gene expression was determined by real time PCR. (B) HIF-1α was induced after treatment of HBSS for 4 h, and then HBSS was changed to complete DMEM or maintained in HBSS with or without 10 μM cycloheximide (CHX). At indicated time points, cell lysates were evaluated for the HIF-1α protein level. (C) [^35^S]Methionine labeled HeLa cells were treated with HBSS or 200 μM CoCl_2_ for 2 or 4 h, and cell lysates were collected and immunoprecipitated by HIF-1α antibody to determine *de novo* protein expression of HIF-1α. (D) HeLa cells were treated with HBSS or hypoxia for 2 h. Polysomal (P) and nonpolysomal (NP) fractions were separated by discontinuous sucrose gradient (10%-50%). The amounts of HIF-1α and β-actin mRNA in polysomal and nonpolysomal fractions were analyzed by reverse transcription-PCR. (E) HeLa cells were treated with HBSS for indicated time points. Total cell lysates were collected and subjected to Western blot analysis. (F) After transfection of pBIC-HIF-1α plasmid, HeLa cells were treated with HBSS for 4 h. CAT and LacZ expression were detected, and the ratio CAT/LacZ represented HIF-1α IRES activity. *p<0.05, indicating significant increase of HIF-1α translation (C), changes of HIF-1α mRNA in polysomal and nonpolysomal fractions (D) and increase of IRES activity by HBSS.

This finding drives us to determine if the cap-dependent translation signaling is induced by HBSS. As shown in Fig. 2E, p70S6K and 4E-BP1 phosphorylation, indexes of cap-dependent translation, however, were significantly inhibited by HBSS. Consistent with the inhibition of cap-dependent translation, Akt phosphorylation, the upstream molecule of mTOR, was also significantly and rapidly inhibited by HBSS. After ruling out the induced HIF-1α by HBSS is related to cap-dependent translation, we next determined if it is through IRES-dependent translation, as it has been reported that 5′ UTR of HIF-1α mRNA contains the IRES structure [13]. IRES activity of HIF-1α was measured by transfection of bicistronic plasmid containing β-gal and CAT, and controlled by CMV and 5′ UTR of HIF-1, respectively. As shown in Fig. 2F, HBSS significantly increased IRES activity of HIF-1α. All these results suggest that nutrient deprivation can induce HIF-1α expression through IRES-dependent translation.

### Beclin 1-independent macroautophagy positively regulates HBSS-induced HIF-1α IRES activity

It has been demonstrated that HIF-1α can be degraded through CMA and proteasome, thus we determined if bafilomycin A1, a lysosome inhibitor, and MG132, a proteasome inhibitor, can accumulate HIF-1α protein in HeLa cells. Indeed as shown in Fig. 3A, both of bafilomycin A1 and MG132 can induce HIF-1 protein accumulation significantly. In addition, the amount of HIF-1α accumulated more by MG132 than by bafilomycin A1 treatment supports the notion that proteasome is the major degradation pathway of HIF-1α. Paradoxically previous findings also suggest that macroautophagy can positively regulate HIF-1α expression despite the underlying molecular mechanism is unknown [27]. Thus to determine the role of macroautophagy in HBSS-induced HIF-1α expression, we first confirmed the ability of HBSS to induce macroautophagy. As shown in Fig. 3B, although HBSS alone cannot significantly induce LC3-II accumulation, it indeed can enhance the response when combined with bafilomycin A1, an index of macroautophagic flux. Next, we used pharmacological and genetic approaches to verify the contribution of macroautophagy in HIF-1 induction caused by HBSS. We found that 3-MA, an inhibitor of class III PI3K leading to the inhibition of macroautophagy [36, 37], can prevent HBSS-induced HIF-1 expression, p62 downregulation and LC3-II accumulation (Fig. 3C). Additionally we found another lysosome inhibitor chloroquine exerts similar effect as bafilomycin A1 (Fig. 3D). Chloroquine alone moderately increased HIF-1α and p62 protein expression, but significantly reversed the effects of HBSS on HIF-1α induction and p62 downregulation.

**Figure 3:** Beclin 1-independent macroautophagy positively regulates HBSS-induced HIF-1α IRES activity in HeLa cells (A) HeLa cells were treated with HBSS, 100 nM bafilomycin A1 or 20 μM MG132 for indicated time points. Total cell lysates were collected and subjected to Western blot analysis. (B-D, H) HeLa cells were treated with HBSS in the absence or presence of 100 nM bafilomycin A1 (B, C), 10 mM 3-MA (C), 100 μM chloroquine (D) or 500 nM rapamycin (H) for indicated time points. Total cell lysates were collected and subjected to Western blot analysis using the indicated antibodies. (E, F, G) After silence of ATG5 (E, F) or Beclin 1 (G) for 72 h, HeLa cells were treated with HBSS for 2 or 4 h. Total cell lysates were collected and subjected to Western blot analysis. (I, J) After silence of ATG5 or Beclin 1, HeLa cells were treated with HBSS for 4 h to determine the HIF-1α gene expression (I) or transfected with pBIC-HIF-1α plasmid for 24 h and then treated with HBSS for 4 h to determine the IRES activity (J). *p<0.05, indicating significant inhibition of HBSS-induced IRES activity.

To exclude the possibility of non-specific effects of 3-MA and chloroquine, we further used siRNA approach to explore the role of macroautophagy in HBSS-induced HIF-1α expression. As a result our data revealed that silence of ATG5 can reverse HBSS-induced HIF-1α expression in HeLa cells (Fig. 3E). To eliminate the off target effect of single si-ATG5 used, we used additional three si-ATG5 RNAs which target different sequences of ATG5 to strengthen confidence in this result. As shown in Fig. 3F, all si-ATG5 RNAs can significantly inhibit HBSS-induced HIF-1α expression. Notably, silence of Beclin 1 failed to affect HBSS-induced HIF-1α expression (Fig. 3G). Considering mTOR inhibition leads to macroautophagy and the ability of HBSS to inhibit Akt/mTOR signaling, we used mTOR inhibitor rapamycin to check the role of mTOR inhibition in HIF-1α expression. As a result rapamycin treatment exerted a rapid p70S6K inactivation as HBSS, however, compare to the control, rapamycin had no significant effect on HIF-1α expression (Fig. 3H). Furthermore, our data revealed no significant changes of HIF-1α mRNA level by si-ATG5 and si-Beclin 1, confirming si-ATG5-reversed HIF-1α expression is not because of the inhibition of HIF-1α mRNA (Fig. 3I). Consistent to the effects on HIF-1α protein expression, silence of ATG5 significantly suppressed HIF-1α IRES activity, while silence of Beclin 1 had no effect (Fig. 3J). All these results suggest that the Beclin 1-independent macroautophagy is involved to upregulate HIF-1α IRES translation under starvation stress.

To understand if above findings observed in nutrient-deprived HeLa cells are cell types specific, we further determined the effects in A431 and A375 cells. Like in HeLa cells, in condition of lysosomal function impairment, HBSS can increase LC3 conversion in A431 and A375 cells (Fig. 4A). Moreover, p62 downregulation under HBSS treatment was restored by chloroquine (Fig. 4A). Next, HBSS also induced significant HIF-1α protein expression in A431 and A375 cells, and this effect can be reversed by 3-MA (Fig. 4B) and si-ATG5 (Fig. 4C). Accordingly HBSS increased HIF-1α IRES activity in A431 and A375 cells (Fig. 4D). These results further suggest that macroautophagy involving in HIF-1α expression through the IRES translation pathway is not cell type-specific.

**Figure 4:** Beclin 1-independent macroautophagy also positively regulates HBSS-induced HIF-1α IRES activity in A431 and A375 cells (A, B) A431 or A375 cells were treated with HBSS in the absence or presence of 100 M chloroquine (A) or 10 mM 3-MA (B) for indicated time points. Total cell lysates were collected and subjected to Western blot analysis. (C) After silence of ATG5 for 72 h, A431 or A375 cells were treated with HBSS for indicated time points. Total cell lysates were collected and subjected to Western blot analysis. (D) As described in Fig. 3I, HIF-1α IRES activity was determined after 4 h treatment with HBSS. *p<0.05, indicating significant increase of IRES activity by HBSS.

### Hypoxia-induced HIF-1α expression also is partially through IRES activation and dependent on Beclin 1 but not ATG5

Since si-ATG6 has been shown to inhibit hypoxia-induced HIF-1α [27], we interested to understand if macroautophagy also plays a role in hypoxia-induced HIF-1 expression through IRES activation. Our data revealed that HIF-1α expression induced by hypoxia was inhibited by 3-MA (Fig. 5A). Notably unlike HBSS, hypoxic effect on HIF-1α protein expression was not changed by si-ATG5 (Fig. 5B), but was reduced by silence of Beclin 1 (Fig. 5C). To eliminate the off target effect, we used three si-Beclin 1 RNAs which target different sequences of Beclin 1 to strengthen confidence in this result. As shown in Fig. 5D, all si-Beclin 1 RNAs partially reversed hypoxia-induced HIF-1α expression. The inhibition of hypoxia-induced HIF-1α protein expression by si-Beclin 1 was not because of interfering with HIF-1α mRNA (Fig. 5E). Interestingly we detected the ability of hypoxia to increase HIF-1α IRES activity, and this action in agreement with protein effect was inhibited by si-Beclin 1 but not by si-ATG5 (Fig. 5F). All these results suggest that hypoxia-induced HIF-1α expression is partial dependent on macroautophagy-associated IRES activity. However, different from nutrient starvation it is through Beclin 1-, but not ATG5-, dependent pathway.

**Figure 5:** ATG5-independent macroautophagy positively regulates hypoxia-induced HIF-1α (A) HeLa cells were cultured under hypoxia condition with or without 10 mM 3-MA for 2 or 4 h. Total cell lysates were collected and subjected to Western blot analysis. (B-D) After silence of ATG5 (B) or Beclin 1 (C, D), HeLa cells were cultured under hypoxia condition for 2 or 4 h. Total cell lysates were collected and subjected to Western blot analysis. In some experiments, HeLa cells were cultured under hypoxia condition for 4 h to determine the HIF-1α gene expression by PCR (E) or transfected with pBIC-HIF-1α plasmid and cultured under hypoxia condition for 4 h to determine the IRES activity (F). *p<0.05, indicating significant inhibition of HBSS-induced IRES activity.

### ROS, AMPK and JNK mediate HBSS-induced HIF-1α expression

Our previous study showed that HBSS induces reactive oxygen species (ROS) production followed by AMPK activation and macroautophagy [29]. Since macroautophagy induction contributes to HIF-1α expression, we determined if ROS/AMPK signaling is also involved in HIF-1α expression under starvation. As a result, ROS scavenger NAC abrogated HBSS-induced HIF-1α expression (Fig. 6A) and macroautophagy (Fig. 6B). Similarly AMPK inhibitor compound C also significantly inhibited HBSS-induced HIF-1α expression (Fig. 6A) and macroautophagy (Fig. 6B). These results demonstrated that ROS/AMPK signaling is involved in HBSS-induced macroautophagy and HIF-1α expression. In addition to ROS/AMPK signaling, nutrient starvation-induced JNK activation has also been shown to induce macroautophagy by phosphorylation of Bcl-2 to interfere with the interaction of Bcl-2 and Beclin 1 [38]. Here we determined if JNK is involved in HBSS-induced HIF-1α expression. As a result, JNK inhibitor SP600125 significantly suppressed HBSS-induced HIF-1α expression (Fig. 6A) and autophagy (Fig. 6B). The findings that inhibition of the upstream molecules of macroautophagy all interferes with HBSS-induced HIF-1α expression further confirmed the important role of macroautophagy in regulation of HIF-1α expression. Furthermore, we determined if ROS/AMPK are the upstream molecules of JNK. We found that NAC and compound C had no significant effects on HBSS-induced JNK phosphorylation (Fig. 6C), but can suppress HIF-1α IRES activity. Moreover, Iressa, as the control inhibitor, did not have significant effect on HIF-1α IRES activity (Fig. 6D). Likewise, JNK inhibitor SP600125 also can suppress HIF-1α IRES activity (Fig. 6D). All these results suggest that ROS/AMPK and JNK are bifurcated signaling cascades triggered by HBSS, and contribute to macroautophagy-dependent HIF-1α IRES activation.

**Figure 6:** ROS, AMPK and JNK are involved in HBSS-induced HIF-1α expression (A, C) HeLa cells were treated with HBSS for the indicated time periods, either in the presence or absence of NAC (10 mM), Compound C (10 μM) or SP600125 (10 μM). Total cell lysates were collected and subjected to Western blot analysis. (B) After treated with NAC (10 mM), Compound C (10 μM) or SP600125 (10 μM) for 30 min, HeLa cells were treated with HBSS with or without 100 nM bafilomycin A1 for the indicated time periods. Total cell lysates were collected and subjected to Western blot analysis. (D) HIF-1α IRES activity was determined after treatment of HBSS for 4 h with or without NAC, Compound C, SP600125 or Iressa (1 μM). *p<0.05, indicating significant inhibition of HBSS-induced IRES activity.

### p38 also positively regulates HBSS-induced HIF-1α expression

It has been demonstrated that inhibition of Akt leads to induce the IRES-dependent translation of cyclin D1 and c-myc through p38 dependent pathways [39]. Here we also found that HBSS significantly inhibited Akt activation (Fig. 2E) but induced p38 activation (Fig. 7A). To understand if p38 phosphorylation plays a role in HBSS-induced HIF-1α expression and macroautophagy, HIF-1α protein level was detected after inhibition of p38. As shown in Fig. 7B and 7C, SB203580, a well defined p38 inhibitor, significantly blocked HBSS-induced HIF-1α expression and IRES activity. However, inhibition of p38 did not have significant effect on macroautophagy (Fig. 7D). Considering above findings that ROS/AMPK signaling is involved in HBSS-induced HIF-1α expression, we further determined if ROS/AMPK is the upstream signaling of p38. As shown in Fig. 7E, inhibition of ROS and AMPK by NAC and compound C, respectively, reduced HBSS-induced p38 phosphorylation. Considering that stimuli-triggered autophagy may also induce ER stress and subsequent p38 activation by IRE-1 signaling pathway [40], we tested if HBSS-induced p38 is related to activation of IRE-1. By detection of the splicing form of XBP1 mRNA which is the IRE-1 downstream signaling [41], we demonstrated that HBSS has no significant effect on XBP1 splicing while thapsigargin which is the well-known ER stressor significantly induced splicing form of XBP1 (Fig. 7F). In that case, we rule out the possibility that HBSS induced p38 is through IRE-1. All these results suggest that ROS and AMPK are the upstream signaling molecules of p38, and p38 enhances HIF-1α IRES activity and subsequent HIF-1α expression through a macroautophagy-independent pathway.

**Figure 7:** p38 mediates HBSS-induced HIF-1α expression independent of macroautophagy (A-F, H) HeLa cells were treated with HBSS in the absence or presence of SB203580 (10 μM) (B-D), bafilomycin A1 (100 nM) (D), NAC (10 mM) (E), Compound C (10 μM) (E), thapsigargin (1 μM) (F), CPG57380 (25, 50 or 100 μM) (H) for indicated time points. Total cell lysates were collected and subjected to Western blot analysis. (G, I) After transfection of constitutively active Akt for 24 h (G) or silence of PTB1 for 72 h (I), HeLa cells were treated with HBSS for indicated time points. Total cell lysates were collected and subjected to Western blot analysis. In (C), HIF-1α IRES activity was determined after treatment of HBSS for 4 h. *p<0.05, indicating significant inhibition of HBSS-induced IRES activity by SB203580.

Next, we wondered if Akt inhibition also mediates the HBSS-induced HIF-1α expression. Since HBSS inhibited Akt phosphorylation, we over-expressed constitutively active Akt to determine the HIF-1α expression under HBSS treatment. As a result, overexpression of constitutively active Akt did not reverse HBSS-induced HIF-1α expression (Fig. 7G). In addition, it has been proved that p38 associated c-myc IRES activity in rapamycin-treated multiple myeloma cells is MNK1 dependent [42]. By using MNK1 inhibitor CGP57380, we determined if this mechanism is involved in HBSS-induced HIF-1α expression. As shown in Fig. 7H, CGP57380 only partially inhibited HBSS-induced HIF-1α expression at 4 h, however, MNK1 phosphorylation which represents for its active form was inhibited under HBSS treatment. In that case, we rule out the contribution of MNK1 in HBSS-induced HIF-1α expression. Finally, since PTB1, an IRES transacting factor (ITAF), has been reported to stimulate IRES-mediated HIF-1 translation during hypoxia [43], we further used siRNA approach to explore its role in our study. As a result our data revealed that silence of PTB1 did not reverse HBSS-induced HIF-1α expression (Fig. 7I).

## DISCUSSION

In this study, we for the first time demonstrate the effect of macroautophagy on HIF-1α expression, and unravel that unlike growth factors-elicited cap-dependent translation and hypoxia-elicited stabilization of HIF-1α, starvation-induced HIF-1α expression is through cap-independent translation mechanism involving Beclin 1-independent macroautophagy. Such Beclin 1-independent macroautophagy controlled-translational process under starvation stress requires ROS/AMPK and JNK signaling. Furthermore, hypoxia also induces cap-independent HIF-1α protein translation, which is controlled by macroautophagy. However, unlike starvation, it is Beclin 1-dependent, but ATG5-independent macroautophagy involved to regulate hypoxia-induced HIF-1α. In addition, p38 also plays an important role in starvation-induced HIF-1α expression (Fig. 8).

**Figure 8:** Schematic summary of nutrient deprivation- and hypoxia-induced HIF-1α expression HBSS starvation induces HIF-1α protein expression through enhancement of IRES activity which is positively regulated by Beclin 1-independent macroautophagy. The Beclin 1-independent macroautophagy is controlled by ROS/AMPK and JNK signaling pathways. Furthermore, p38 which is activated by ROS-mediated AMPK also positively regulates HBSS-induced HIF-1α IRES activity but in a macroautophagy-independent manner. In addition, hypoxia not only stabilizes HIF-1α through inhibition of proteasome degradation pathway, but also induces IRES activity through an ATG5-independent macroautophagy pathway.

HIF-1α is a transcription factor that has been reported to control more than 60 genes and has been demonstrated to play an important role in tumor angiogenesis, metastasis, growth and chemoresistance [44-46]. Our present study shows that in addition to hypoxia, starvation, another environmental phenomenon in solid tumors, can also induce HIF-1α expression. Thus HIF-1α is suggested to play a crucial role in tumorigenesis under starvation condition. In addition, HBSS-induced HIF-1α was reduced at 6 h, and it may be due to cell apoptosis as demonstrated in our previous work [29]. Notably although extent of HIF-1α expression induced by starvation is much less than that induced by hypoxia, both responses display a synergistic effect, suggesting the differential molecular mechanisms for HIF-1α induction by the two solid tumor-harboring metabolic microenvironments. Moreover, starvation also can induce HIF-1α expression in HUVEC as well as in various cancer cell types examined, indicating that this effect is a general action, and not specific to cancer cells only. In addition, our previous work demonstrated that HBSS can induce ROS production within 30 min [29]. In the present study, cysteine, a precursor of glutathione [47], can reverse HBSS-induced HIF-1α expression, implying that ROS is involved in starvation-induced HIF-1α expression, and our NAC result indeed supports this notion.

Unlike hypoxia-induced HIF-1α majorly by inhibition of HIF-1α protein degradation via proteasome system, the enhancement of HIF-1α mRNA binding to polysome by HBSS indicates that starvation induces HIF-1α expression through enhancement of translation. Unlike cytokines and EGF, which induce HIF-1α by Akt/mTOR-dependent translation [48], starvation deficient of growth factors inhibits Akt and mTOR downstream signaling including 4E-BP1 and p70S6K phosphorylation. Our data further show that starvation-induced HIF-1α expression is through IRES-dependent translation. In this aspect, it has been demonstrated that serum starvation can induce HIF-1α IRES activity [13]. In the present study, using reporter assay containing human HIF-1α 5′UTR [35], we demonstrate the increased HIF-1α IRES activity under HBSS starvation. The results of hypoxia are different from starvation; hypoxia induces HIF-1α IRES activity but has no significant effect on the mRNA binding to polysome. These paradoxical data on HIF-1α regulation by hypoxia might be because of the inhibition of cap-dependent translation, but the increased IRES-translation as reported previously [13].

It is well known that CMA is an additional pathway besides proteasome system to degrade HIF-1α protein [26-28]. By comparing the effects of lysosome and proteasome inhibitors on HIF-1α accumulation, we found that MG132 treatment can accumulate more HIF-1α protein than bafilomycin A1. In addition, another lysosome inhibitor chloroquine also can induce HIF-1α accumulation, further supporting the notion that HIF-1α can be degraded through a lysosome-associated pathway. In our study we found the ability of HBSS to induce macroautophagy, but such stress-conferred protein degradation pathway seems not to regulate the protein stability of induced HIF-1α. Instead it is interestingly to note that macroautophagy is involved to positively regulate starvation-induced HIF-1α expression. Moreover, such event is also applied in the case of hypoxia-induced HIF-1α expression. Furthermore, there are conventional and alternative macroautophagy pathways [17]. Of the alternative pathway, Beclin 1-independent macroautophagy can be induced by different stresses [19, 22, 24, 25]. Our data demonstrate that si-ATG5 but not si-Beclin 1 significantly reverses starvation-induced HIF-1α expression. Conversely, si-Beclin 1 rather than si-ATG5 inhibits the response induced by hypoxia. Thus, it is suggested that the alternative macroautophagy is an essential event to trigger HIF-1α IRES activity in cells facing different stresses like nutrient starvation and hypoxia. However, currently it remains unknown how alternative types of macroautophagy with independence on either ATG5 or Beclin-1 and relying on stress context are differentially regulated, but mediate the same effect on increasing HIF-1α IRES activity. Considering that Beclin 1 interacts with Class III PI3K to induce macroautophagy formation, some papers demonstrated that 3-MA, a well-known Class III PI3K inhibitor, cannot interfere with Beclin 1-independent macroautophagy-induced effect [22, 23]. However, 3-MA has also been reported to inhibit Beclin 1-independnt macroautophagy-induced cell death induced by staurosporine [25] as our finding in starvation condition. Thus we propose that Class III PI3K might be involved in macroautophagy formation in a Beclin 1-independent manner. In that case, we suggest that the underlying mechanism of alternative macroautophagy formation is more complicated than we expect.

After showing the role of alternative macroautophagy in starvation-induced HIF-1α expression, and knowing the crucial function of mTOR inhibition on macroautophagy initiation, we consider the contribution of mTOR signaling inhibition induced by nutrient starvation in HIF-1α upregulation. Using rapamycin which is a specific mTOR inhibitor, our results show its inability to induce HIF-1α expression. Thus, we conclude that it is not mTOR inhibition alone but requiring other signaling pathways and molecular events concomitantly provided by starvation to induce HIF-1α IRES activity.

Finally, unlike well-studied mTOR signaling in the cap-dependent translation, the mechanism for IRES-mediated protein translation is unclear. Our results demonstrate that Beclin 1-independent macroautophagy can positively regulates starvation-induced HIF-1α IRES translation. However, how macroautophagy regulates HIF-1α IRES translation needs to be further studied. Considering that the important function of macroautophagy is to recycle proteins to provide amino acids and fatty acids to mitochondrial energy production under starvation condition [49], we suggest that macroautophagy functions through at least two possible mechanisms to control starvation-induced HIF-1α IRES translation. One is degradation of molecules which inhibited HIF-1α IRES translation under normal condition. Another is recycling proteins to release amino acids and fatty acids to provide mitochondria energy production for HIF-1α IRES translation. In the case of hypoxia, silence of ATG6 has been reported to inhibit hypoxia-induced HIF-1α [27], implying that macroautophagy may positively regulate hypoxia-induced HIF-1α expression. Our results also support this notion and further demonstrate that it is through ATG5-independent macroautophagy, an alternative autophagy [18]. Finally, according to our HBSS and hypoxia results, we for the first time demonstrate that Beclin 1- and ATG5-independent autophagy positively regulate HBSS- and hypoxia-induced HIF-1α, respectively.

Akt and p38 have been demonstrated to regulate IRES-dependent protein translation, however, the role in regulation of IRES activity is more ambiguous. For example, inhibition of Akt and p38 reduce TNF-α-induced IRES-dependent HIF-1α translation [14]. In contrast, inhibition of Akt activity induces IRES-dependent translation of cyclin D1 and c-myc through p38-dependent pathway [39]. Despite the conflict role of Akt in IRES activity observed in previous studies, p38 seems to be a positive regulator in this effect. In the present study we showed that p38 can positively regulates starvation-induced HIF-1α translation, while Akt activity does not have significant effect on starvation-induced HIF-1α translation. Moreover, since p38 are not involved in starvation-induced macroautophagy formation, the mechanism of p38 regulation of starvation-induced HIF-1α IRES activity and protein expression is needed to be further investigated. Interestingly, ROS and AMPK are involved in starvation-induced p38 phosphorylation. It has been reported that AMPK can active p38 through a TAK1 dependent pathway [50]. Although ROS-AMPK-p38 signaling cascade has been demonstrated to induce apoptosis, glucose uptake and cyclooxygenase-2 expression [51, 52], we for the first time link this pathway to IRES activity.

In summary, HIF-1α is an important protein to regulate tumorigenesis. In the present study, we demonstrate a novel mechanism responsible for nutrient starvation-induced HIF-1α expression. This mechanism is through Beclin 1-independent macroautophagy to increase IRES-dependent HIF-1α translation. Furthermore, ATG5-independent macroautophagy also can positively regulate the hypoxic-mediated cap-independent protein translation of HIF-1. Thus, it is a novel finding in this study to expand the multiple functions of macroautophagy under stress conditions to positively control the protein translation through cap-independent pathway.

## MATERIALS AND METHODS

### Cell culture

HeLa, A431 and A375 cells were obtained from the American Type Culture Collection. HeLa, A431 and A375 were cultured in Dulbecco's modified Eagle medium (Invitrogen) complete medium supplemented with 10% (v/v) heated-inactivated fetal bovine serum (Biological Industries). Human umbilical vein endothelial cells (HUVEC) were purchased from ScienCell (Carlsbad, CA, USA). For hypoxic treatment, cells were placed into a hypoxic chamber with an oxygen environment lower than 1%.

### Reagents

HBSS (Invitrogen) contain 5 mM glucose, 1.26 mM CaCl_2_, 0.493 mM MgCl_2_, 0.407 mM MgSO_4_, 5.33 mM KCl, 0.441 mM KH_2_PO_4_, 4.17 mM NaHCO_3_, 137.93 mM NaCl, and 0.338 mM Na_2_HPO_4_. Bafilomycin A1, CGP57380, CoCl_2_, Compound C, Cycloheximide, SB203580 and SP600125 were from Calbiochem. 3-Methyladenine (3-MA), chloroquine, N-acetyl-cysteine, rapamycin and other chemicals were obtained from Sigma Aldrich. Iressa was from Cayman Chemical Company (Ann Arbor, MI, USA). The anti-HIF-1α (for immunoblot) and Beclin 1 antibodies were from Becton Dickinson. Antibodies specific to phosphorylated JNK, p38, Akt, p70S6K (Thr389), 4E-BP1 (Ser65), p62, total Akt, p70S6K and 4E-BP1 were from Cell Signaling. Antibodies specific to HIF-1α (for immunoprecipitation), PTB1, p38, JNK and normal rabbit IgG were from Santa Cruz. The anti-ATG5 antibody was from Abcam. The anti-LC3 antibody was from MBL. The anti-β-actin antibody was from Merck Millipore. All siRNAs and DharmaFECT Transfection Reagents were from Dharmacon. [^35^S]Methionine was purchased from GE Heathcare.

### Quantitative real-time PCR

The cells were harvested using TriPure reagents (Roche) and total RNA was extracted by following the manufacturer's protocol. cDNAs were synthesized by using MMLV reverse transcriptase (Promega) and PCR was performed by using FastStart SYBR Green Master (Roche) and ABI Prism 7900 (Applied Biosystems). Each PCR reaction contained the cDNA, the Master Mix, and the following primers: HIF-1α (forward: 5′- TGCTCATCAGTTGCCACTTC -3′, reverse: 5′- TCCTCACACGCAAATAGCTG -3), and β-actin (forward: 5′- CGGGGACCTGACTGACTACC -3′, reverse: 5′- AGGAAGGCTGGAAGAGTGC -3′).

### de novo translation

HeLa cells were cultured with methionine-free DMEM containing dialysed FBS for 2 h, and then 1 mCi [^35^S]methionine was added for 30 min. After starvation by HBSS or CoCl_2_ treatment, cells were lysed with RIPA buffer and precleaned with normal IgG. Immunoprecipitation was performed by HIF-1α antibody. Immunoprecipitated protein complexes were subjected to electrophoresis and expose to x-ray film.

### Polysome analysis

Polysome analysis was conducted as described [53]. Briefly, cycloheximide was added 30 min before HeLa cells were collected. Cells were scraped, resuspended with RSB buffer (10 mM Tris-HCl at pH 7.4, 10 mM NaCl, 3 mM MgCl_2_ and 1000 U/ml RNasin) and lysed in equal volume of polysome extraction buffer (RSB buffer containing 1% Triton X-100, 1% deoxycholate, and 2% Tween 20). After centrifuging, the cell extract was layered onto a 4 ml discontinuous 10% to 50% sucrose gradient. Fractionation was obtained with centrifugation at 36,000 rpm for 2 h at 4℃, in a Beckman SW50 rotor. The gradient was monitored at 254 nm with ISCO UA-6 absorbance detector. The polysomal and nonpolysomal fractions were separated and subjected to mRNA isolation. cDNA was synthesized from equal volume of fractionated RNA and then PCR was performed with the following primers: HIF-1α (forward: 5′- CTGGATGCTGGTGATTTGGA -3′, reverse: 5′- TTCATATCCAGGCTGTGTCG -3′) and β-actin (forward: 5′- GCTGGAAGGTGGACAGCGAG-3′, reverse: 5′- TGGCATCGTGATGGACTCCG -3′). The PCR products were separated on a 3% agarose gel and quantified by ImageJ.

### *Xbp-1* splicing

*Xbp-1*splicing was analyzed by reverse transcription-PCR with the following primers: *Xbp-1* (forward: 5′- GAGTTAAGACAGCGCTTGGG -3′, reverse: 5′- ACTGGGTCCAAGTTGTCCAG -3′) and β-actin (forward: 5′- GCTGGAAGGTGGACAGCGAG -3′, reverse: 5′- TGGCATCGTGATGGACTCCG -3′). The PCR products were separated on a 9% acrylamide gel and quantified by ImageJ.

### Plasmids transfection

The constitutive active Akt plasmid was kindly provided by Dr. Bing-Chang Chen (School of Respiratory Therapy, College of Medicine, Taipei Medical University, Taiwan). The pBIC-HIF-1α [35] plasmid was a gift from Dr. Martin Holcik (Children's Hospital of Eastern Ontario Research Institute, Canada). Plasmids were transfected by Lipofectamine 2000 (Invitrogen) according to the manufacturer's instructions.

### IRES activity assay

IRES activity was assayed by bicistronic reporter plasmid pBIC-HIF-1α contains 2 to 352 bp of human HIF-1α 5′UTR which has been ruled out the possibility of cryptic promoter activity and splicing of the bicistronic mRNA. Cells were transfected with pBIC-HIF-1α. After indicated treatment, the amount of chloramphenicol acetyltransferase (CAT) was determined by CAT ELISA (Roche) according to the manufacturer's instructions. β-Galactosidase (β-Gal) enzymatic activity was determined by spectrophotometric assay using *o*-nitrophenyl-β-D-galactopyranoside. The relative IRES activity was calculated as the CAT/β-Gal ratio.

### Immunoblot analysis

Protein expression was determined in cell lysates by electrophoresis and immunobloting as we previously described [29].

### Statistical evaluation

Values were expressed as the mean±S.E.M. of at least three independent experiments. An analysis of variance (ANOVA) was used to assess the statistical significance of the differences, and *p* values of < 0.05 were considered statistically significant.
